RETRACTED

# lncRNA GAS5 Induces Cell Apoptosis in Acute Myeloid Leukemia by Targeting Nrf2

**DOI:** 10.1155/2022/5178122

**Published:** 2022-08-24

**Authors:** Xiaohua Qin, Yanling Jiang, Xiaojun Zhang, Dan Li

**Affiliations:** Department of Hematology, Huizhou Central People's Hospital of Guangdong Province, China

## Abstract

**Objective:**

This study is aimed at investigating the molecular mechanism of lncRNA GAS5-induced cell apoptosis in acute myeloid leukemia (AML) by targeting Nrf2.

**Methods:**

The RNA interfering technique was utilized to silence THP-1 in AML cell line, and lncRNA GAS5 expression in cell line was determined by real-time PCR. EdU experiment and flow cytometry were used to detect the apoptosis and proliferation ability of cells in different groups. PD-L1, STAT3, AKT, and MMP9 expressions were determined by Western blot.

**Results:**

The si-RNA significantly inhibited the expression of lncRNA GAS5 in THP-1 cells. Compared with the si-NC group, the difference in cell apoptosis between lncRNA GAS5 and Nrf2 groups was significant (*P* < 0.05). Compared with the lncRNA GAS5 group, the number of apoptotic cells in the lncRNA GAS5+Nrf2 group significantly reduced (*P* < 0.05). Compared with the si-NC group, the differences in the levels of four proteins between lncRNA GAS5 and Nrf2 groups were significant (*P* < 0.05). In lncRNA GAS5+Nrf2 and lncRNA GAS5 groups, PD-L1 expression increased, while the expression of STAT3, AKT, and MMP9 decreased.

**Conclusion:**

In AML cells, lncRNA GAS5 with Nrf2 could regulate the proliferation and apoptosis of AML cells. lncRNA GAS5 inhibited Nrf2 expression, regulated cell apoptosis and proliferation, and further inhibited the progression of AML disease.

## 1. Introduction

Acute myeloid leukemia (AML) is a disease common in adults and older adults. The proportion of patients 65 years and older was 54 percent [1, 2]. AML, which originates from a small number of leukemic stem cells in the body, is a malignant tumor of the heterogeneous hematopoietic system and is characterized by the clonal proliferation of progenitor cells in peripheral blood, bone marrow, and tissues [3, 4]. AML is a common malignant tumor in the blood system. Unlike other karyotype tumors, AML often carries multiple characteristic types of genetic abnormalities that not only contribute to the development of AML disease but also affect disease progression and outcome [5, 6]. For example, the ability to invade and infiltrate tissue and the ability of cells to proliferate affect the clinical presentation of patients in different ways [7]. Chemotherapy and supportive care for AML are still evolving. Symptoms improved or relieved in some patients. However, relapses can still occur. According to relevant studies, the overall 5-year survival rate is only 40% to 50% [8]. Research on specific targeting of leukemia stem cell therapy is beneficial to reduce disease recurrence and even disease recovery. Therefore, it is necessary to continue research on targeted therapy for AML.

RETRACTED

In a basic biological process, long noncoding RNA (lncRNA) plays a very important regulatory role. Once the disorder occurs, human internal disease will be caused. A clear understanding of the biological characteristics of lncRNA can get more different insights into pathogenic mechanism, which is beneficial to better understanding the occurrence of disease and getting more opportunities of diagnosis and treatment [9, 10]. lncRNA growth arrest-specific transcript 5 (lncRNA GAS5) is correlated with the pathogenesis of many diseases, and its expression level and clinical pathological features are both associated with patient prognosis to some extent. The expression of lncRNA GAS5 in multiple tumors is low, and it acts as a tumor-suppressor gene. Some studies reveal that lncRNA GAS5 can inhibit the proliferation of multiple cells and promote their apoptosis, and the action mechanism of these cells forms the basis of tumor inhibition together [11, 12]. Yunusov et al. [13] showed in their study that lncRNA expression demonstrated tissue specificity and cell specificity as well as the specificity of eukaryote at developmental stage. lncRNA GAS5 is a member of lncRNA and plays a regulatory role in the development of many acute and chronic diseases. Besides, regulatory proteins with transcriptional function with lncRNA GAS5 adjust the activation or inhibition of relevant gene transcription by titration [14, 15]. Li et al. [16] confirmed that lncRNA GAS5 get involved in the differentiation of stroma stem cells and acted as a regulator. Nuclear factor erythroid 2-related factor 2 (Nrf2) is a key transcription factor in the fundamental expression of oxidative stress. It exists in multiple body organs and promotes cell apoptosis, inflammation, autophagy, oxidative stress, heterologous biological metabolism, and the gene expression of cellular bioenergy. Loss of Nrf2 or activation disorder results in the change in the sensitivity of stimulus corresponding to cells [17, 18]. Nrf2 contains a highly conservative basic leucine zipper structure, which plays an important role in protecting body against the damage caused by allogenic substances and oxidative stress. The role of Nrf2 in carcinogenesis includes two aspects. One is the prevention of cancer for healthy people, and another is the positive effect of the abnormal persistent activity of Nrf2 on carcinogenesis [19].

RETRACTED

In this study, the targeted induction of Nrf2 was used to explore the mechanism of lncRNA GAS5 in AML cell apoptosis, in order to more comprehensively and effectively understand the mechanism of lncRNA GAS5 in AML disease and further provide reference for the disease control and targeted therapy of AML.

## 2. Materials and Methods

### 2.1. Reagents

Main reagents included leukemia cell strains HL-60 and THP-1 (Guangzhou Sagene Biotech Co., Ltd.), sheep anti-human NQO1 antibody (1 : 1,1000, Santa Cruz, USA), Lipofectamine 2000 (Invitrogen), rabbit anti-human Nrf2 antibody (1 : 1000, ABZOOM, USA), fetal calf serum (Israel BIOIND Company), Western and IP lysate (Beyotime Biotechnology Co., Ltd.), and Nrf2 si-RNA which were obtained from 5′-AAG AGT AGC TGG AAA AAC-3′ from GenePharma (Shanghai, China).

### 2.2. Cell Grouping and Transfection

The transfection was performed by using the Lipofectamine 2000 kit (Invitrogen, USA) according to the instructions, and the cells were divided into negative control si-RNA (si-NC) group, lncRNA GAS5 plasmid (overexpressed lncRNA GAS5 was transfected) group, Nrf2 group (Nrf2 interfering plasmid was transfected), and lncRNA GAS5+Nrf2 group (overexpressed lncRNA GAS5 and Nrf2 interfering plasmid were transfected). The upstream and downstream primers of lncRNA GAS5 were 5′-TGGATTTCGTGGCCCCAGTGCTA-3′ and 5′-TTCATCCTGTTCTTCCTCGGCG-3′, respectively. The primers of negative control group were 5′-ACAGAGCCTCGCCTTTGCCGAT-3′ and 5′-CTTGCACATGCCGGAGCCGTT-3. The primers of si-RNA-1 were 5′-TGACGGCGAGGACAGAGGAG-3′ and 5′-CCCAGAGGGCAGCCATAGTG-3. The primers of si-RNA-2 were 5′-CCCACAACAUGAAAGAAACTT-3′ and 5′-AUUUCUUUCAUGUUGUGGGrl-3. The culture medium was replaced with the one without antibiotic 1 hour after transfection. The RNA level was determined 48 hours post transfection.

### 2.3. Detection of Cell Proliferation by EdU Staining

EdU was utilized to detect cell proliferation. EdU solution was diluted in a ratio of 1000 : 1 in cell culture medium, and appropriate amount of 50 *Μ*m EdU culture medium was prepared. If the incubation lasted for less than 2 hours, EdU with a concentration of 10 to 50 *μ*M should be selected. If the incubation lasted for more than 24 hours, EdU with a concentration of 1-0 *μ*M should be selected. The preservation time of the prepared culture medium depended on its nature. 100 *μ*L 96-pore plate EdU culture medium and 100 *μ*L staining reaction fluid were selected. Cells should be immersed in the EdU culture medium. A continuous supply of nutrients should be guaranteed during the EdU incubation period. Cell were rinsed with phosphate buffer saline (PBS) once or twice (5 minutes per time) to remove uninfiltrated EdU of DNS. Most cell lines were incubated for 2 hours. Longer incubation indicated more proliferation. Cells in each group were inoculated into the 96-pore plate through trypsin. After cells were cultured for 24 and 48 hours, they were stained and washed according to the number of reagents. After that, cells were photographed and analyzed by an inverted fluorescence microscope.

RETRACTED

### 2.4. Western Blot (WB)

The cultured cells were extracted, and culture solution was thoroughly absorbed in blotting paper. Next, 3 mL PBS (precooled at 4°C) was added slowly and horizontally and then oscillated for 1 minute gently. After that, cells were rinsed and effluent was discarded. The above steps should be repeated twice. Then, the culture flask with residual fluid removed completely was placed on ice and then added with lysate. 25 *μ*L phenylmethylsulfonyl fluoride (PMSF) (100 mM), 1 mL ristocetin-induced platelet agglutination (RIPA), and 110 *μ*L phosphatase inhibitor (Pi) were selected. The solution was shaken evenly until there was no crystal and then mixed with the lysate completely. Next, it was put into ice. After 100 *μ*L lysis buffer was added, a sterile spatula was used to scrape to one side of the flask. The cells were split on ice for half an hour. During the procedure, the flask needed to be oscillated slowly and gently for 10 minutes so that the cells dissolved completely. After the split, the mixture was transferred to a 1.5 mL centrifuge tube and then centrifuged at 4°C and 12000 rpm for 15 minutes. After that, supernatant was replaced, and protein concentration was detected in the precooled EP tube. Next, gel electrophoresis was performed. After sodium dodecyl sulfate polyacrylamide gel electrophoresis (SDS-PAGE), the polyvinylidene fluoride (PVDF) membrane was transformed and sealed for 2 hours. According to the leukorrhea of proteins, the approximate position of target proteins was determined. The PVDF membrane was cut into the size of a gel block and soaked in methanol for 2 minutes. Filter paper was placed into a membrane transformation clip gently. Sponge, filter paper, separation gel, PVDF membrane, filter paper, and sponge were placed successively. The device was placed in a membrane transformation groove. Then, the precooled buffer solution was added, and the membrane was transformed for 80 minutes at a voltage of 90 V. Next, the PVDF membrane was extracted and rinsed with Tris-buffered saline tween (TBST). After finding the position of proteins, the PVDF membrane was cut. After being soaked in the TBST solution for 3 minutes, the PVDF membrane was sealed at a room temperature for 2 to 3 hours. Then, it was rinsed with the TBST buffer. After that, the primary antibody working liquid was added and incubated overnight at 4°C. The primary antibody was poured out, and then the PVDF membrane was washed with the TBST buffer again. Next, 15 mL secondary antibody working liquid was added and then oscillated at room temperature for 3 hours. After that, the secondary antibody was poured out, and the PVDF membrane was washed with the TBST buffer. The back side of membrane was rubbed with filter paper, and then the membrane was placed in culture medium. The membrane was poured with 1 mL electrochemiluminescence (ECL) white solution and 1 mL ECL black solution with a size of 2 cm × 7 cm and washed about 10 times. The PVDF membrane was dried with filter paper and then wrapped. The coloring solution was added for exposure and development, and fluorescent film sweeper was used for scan.

RETRACTED

### 2.5. Flow Cytometry

Cells were digested with 0.25% pancreatin to excessive digestion. During the digestion, 2% bovine serum albumin (BSA) was added, and 1× PBS or 1× binding buffer was selected to rinse cells to remove ethylenediaminetetraacetic acid (EDTA). 10× binding buffer was diluted into 1× binding buffer with deionized water. Then, cells were collected for 5 to 10 minutes and then centrifuged at 2000 rpm for 5 minutes. Next, cells were rinsed and resuspended with the precooled 1× PBS at 4°C. After that, cells were centrifuged at 2000 rpm for 5 to 10 minutes and then rinsed. The last step of washing was to remove supernatant to avoid PBS residue and effect on experimental results. Then, 300 *μ*L 1× binding buffer suspension cells were added and then mixed with 5 *μ*L Annexin V-FITC evenly. The mixture was kept away from light and incubated at room temperature for 15 minutes. 200 *μ*L 1× binding buffer was added before loading the machine, and 5 *μ*L propidium iodide (PI) was added for staining 5 minutes before loading the machine. Because PI was poisonous, it is necessary to wear glove during use to the absorption of PI by skin. When multiple samples were detected at a time, the interval should range between 30 and 60 s. To avoid fluorescent decay, flow cytometry should be adopted within 1 hour. Long staining time caused the high apoptosis rate, which should be avoided. During Annexin V-FITC staining, PI staining could be added as early as 5 minutes before loading the machine. PI and Annexin V-FITC were both photosensitizing substances. Hence, they should be kept away from light during operation and staining needed to be performed in dark. During incubation stage, the container should be wrapped in drawer or with aluminum foil, and a microscope was used for observation in dark room.

RETRACTED

### 2.6. Detection of mRNA Expression by qRT-PCR

The total RNA was extracted with TRIzol reagent (Invitrogen, USA). The cDNA was synthesized by using the reverse transcription kit (TaKaRa, Japan). The amplification was performed on a ABI 7500 Real-Time PCR system (ABI, USA). The reaction procedure of PCR was set at 95°C for 10 minutes, 95°C for 15 s, 60°C for 30 s with 40 cycles, 72°C for 15 s, 95°C for 15 s, 60°C for 1 minute, and 95°C for 15 s. The U6 was set as the internal reference gene. The primer sequences are shown in Table 1.

### 2.7. Statistical Methods

The statistical analysis was performed by the SPSS 19.0 statistical software (IBM SPSS Statistics, USA). The differences between two groups were analyzed using the independent *t* test. Measurement data were expressed by mean ± standard deviation (SD). Enumeration data were analyzed by the *χ*^2^ test and expressed by percentage (%). All experiments were performed in triplicate. A two-sided *P* value less than 0.05 was set as significant difference.

## 3. Results

### 3.1. Inhibition of lncRNA GAS5 with si-RNAs

As shown in Figure 1, after cells were transfected with si-RNAs, the lncRNA GAS5 level in THP-1 cell line downregulated significantly. Since si-1 showed more robust knockdown effect compared to si-2, si-1 was selected for following experiments.

### 3.2. Influences of lncRNA GAS5 in THP-1 Cell Line on Cell Proliferation

After cell lines were transfected by si-RNA-NC and GAS5 in THP-1 cell line, the detection of cell proliferation is shown in Figure 2. With time prolonging, the cell proliferation in each group gradually increased. Compared with that of si-RNA-NC group, the cell proliferation of si-1 and si-2 groups was inhibited.

### 3.3. Cell Apoptosis Detection Results

Cell apoptosis detection results are displayed in Figure 3. Q2-1 represented necrotic cell area, Q2-2 referred to late apoptotic cells, Q2-3 denoted viable cell area, and Q2-4 represented early apoptotic cell area. Next, the apoptosis rate of the cells in 4 groups was compared quantitatively (Figure 4). Compared with the si-NC group, the difference between the lncRNA GAS5 group and Nrf2 group was remarkable (*P* < 0.05). However, there was no significant difference in the lncRNA GAS5+Nrf2 group (*P* > 0.05). Compared with lncRNA GAS5 group, the number of apoptotic cells in lncRNA GAS5+Nrf2 group apparently reduced (*P* < 0.05).

### 3.4. Influence of lncRNA GAS5 and Nrf2 on Cell Proliferation

As displayed in Figure 5, the difference between lncRNA GAS5 and Nrf2 group was significant compared with the cell proliferation rate in si-NC group (*P* < 0.05) in THP-1 cells. However, there was no remarkable difference in the lncRNA GAS5+Nrf2 group (*P* > 0.05). Compared with the lncRNA GAS5 group, the cell proliferation rate of the lncRNA GAS5+Nrf2 group significantly decreased (*P* < 0.05).

RETRACTED

### 3.5. Influences of lncRNA GAS5 and Nrf2 on Relevant Protein Expressions in THP-1 Cells

As shown in Figures 6 and 7, the protein levels of programmed death ligand-1 (PD-L1), signal transducer and activator of transcription 3 (STAT3), AKT downstream, and matrix metalloproteinase-9 (MMP9) in cells of different groups were determined. Compared with the si-NC group, the contents of 4 proteins between lncRNA GAS5 group and Nrf2 group showed remarkable differences (*P* < 0.05). The expressions of PD-L1 in the lncRNA GAS5+Nrf2 group and lncRNA GAS5 groups increased, while the expressions of protein contents of STAT3, AKT, and MMP9 decreased. The differences were statistically significant (*P* < 0.05). The comparison of protein contents of PD-L1, STAT3, AKT, and MMP9 between lncRNA GAS5 group and Nrf2 group revealed no remarkable difference (*P* > 0.05).

## 4. Discussion

Leukemia is a clonal malignant leukemia transformed in hemopoietic stem cells. AML is a heterogeneous malignant hematologic tumor. Chromosomal translocation is the commonest cause of the malignant transformation of hematopoietic progenitor cells [20]. AML patients suffer mainly from the blocking of normal differentiation and apoptosis of hematopoietic cells, the abnormal proliferation of bone marrow hematopoietic cells, and the accumulation of a large number of immature progenitor cells in the bone marrow peripheral blood. As a result, the function of normal cells is impaired, which results in anemia, hemorrhage, and infection among patients. Among the patients with advanced AML, leukemia metastasizes to the liver, spleen, and other organs, which finally leads to the attenuation of organ functions and death [21]. Nrf2 plays an important role in cancer chemotherapy resistance [22]. Nrf2 expression is associated with tumor mutational load in AML. The frequency of gene mutation and drug resistance of patients with overexpression of Nrf2 is higher [23]. The overexpression of Nrf2 protects AML cells from cytosine arabinoside-induced cell apoptosis in vitro and increases the risk of drug resistance related to gene mutation in body. The overexpressed Nrf2 may get involved in tumor chemotherapy resistance. Previous study [24] indicated that high expression of Nrf2 could induce the instability, dependence, and drug resistance of genes in AML and caused the increase in AML gene mutation frequency, which provided a new strategy for clinical practice. In addition, lncRNA GAS5 was apparently correlated with the prognosis of AML [25]. The correlation coefficient was *P* = 0.018. Increased GAS5 expression increased bone marrow suppression and further led to the poor prognosis of AML. Some studies demonstrated that GAS5 acted as the ribose inhibitor of glucocorticoid receptor (GR), and the abnormal level of GAS5 might change the reaction of hematopoietic cells to glucocorticoid. GAS5 could interact encoded by NR3C1 gene and inhibit its transcriptional activity. Another study verified that GGAT, CGGT, and GGGT haplotypes were associated with a higher AML risk among research objects [26].

RETRACTED

The genetic molecules of lncRNA in oncobiology attract people's attention. lncRNA GAS5 was underexpressed in colorectal cancer, and overexpressed lncRNA GAS5 could regulate histone methyl transferase and body and promote the inhibition or metastasis of cancer [27]. The apoptosis and proliferation rates of cells in four groups were compared. Compared with si-NC group, the difference between lncRNA GAS5 plasmid and Nrf2 group was remarkable (*P* < 0.05). However, there was no significant difference in the lncRNA GAS5+Nrf2 group (*P* > 0.05). Compared with lncRNA GAS5 group, the number of apoptotic cells in lncRNA GAS5+Nrf2 group apparently decreased (*P* < 0.05). The expression of lncRNA GAS5 in AML tissue obviously declined, which suggested that lncRNA GAS5 could inhibit cancer in AML. Unlike cell necrosis, cell apoptosis refers to the maintenance of a stable internal environment and the spontaneous and orderly death of cells controlled by genes. It is an active process involving the activation, expression, and regulation of a series of genes. Cancer genes usually change with the changes in the cells proliferate and grow. The analysis of cell proliferation rate revealed that overexpressed lncRNA GAS5 could inhibit cell proliferation and promote cancer cell apoptosis. Nrf2 was actively expressed in oncogenes. Previous study demonstrated that the downregulation of GAS5 resulted in the upregulation of renal injury pattern induced by sepsis in body [28]. GAS5 reduced cell apoptosis by activating PGC-1aNrf2 pathway. Besides, the overexpression of GAS5 promoted the improvement of survival rate among mice and alleviated renal injury, which suggested that GAS5 expression and Nrf2 targeted induction were correlated with the development of disease to some extent. Based on the expressed lncRNA GAS5, the number of apoptotic cells in lncRNA GAS5+Nrf2 group significantly reduced, which indicated that lncRNA GAS5 could inhibit the expression of Nrf2, control cell apoptosis and proliferation, and further inhibit the progression of AML disease. Matrix metalloproteinase (MMPS) could degrade extracellular matrix and basilar membrane and induce tumor dispersion and metastasis. STATA3 could bind to PD-L promoter region and regulate the high expression of PD-1. Tumor progression was closely related to abnormal cell proliferation and apoptosis. It was demonstrated that the contents of four proteins in lncRNA GAS5 group and Nrf2 group all revealed significant difference compared with si-NC group (*P* < 0.05). The expressions of PD-L1 in lncRNA GAS5+Nrf2 group and lncRNA GAS5 group increased, while the expressions of protein contents of STAT3, AKT, and MMP9 decreased, which showed that lncRNA GAS5 could downregulate Nrf2 expression, activate STAT3 signal pathway, regulate the expressions of AKT and MMP9, and further inhibit cell proliferation and promote cell apoptosis.

RETRACTED

## 5. Conclusion

The regulatory mechanism of lncRNA GAS5 in cell apoptosis in AML disease through targeted Nrf2 induction was discussed. Based on the lncRNA GAS5 expression, the number of apoptotic cells in the lncRNA GAS5+Nrf2 group was remarkably reduced, which demonstrated that lncRNA GAS5 could inhibit Nrf2 expression, control cell apoptosis as well as proliferation, and further inhibit the progression of AML disease. The binding of lncRNA GAS5 with Nrf2 transcription factor helped better understand the prevention mechanism of AML and provided potential biomarker for the study on AML to reduce the recurrence of AML and prolong patient survival. In future research, AML development mechanism should be investigated based on the specific regulatory methods of lncRNA GAS5 for the transcriptional activity of IGF1R promoter from multiple perspectives to provide some ideas and experimental support for the rehabilitation of AML patients.

## Figures and Tables

**Figure 1:** Results of lncRNA GAS5 level knockdown by si-RNAs.

**Figure 2:** Curves of cell proliferation.

**Figure 3:** Flow cytometry in each group in THP-1 cells.

**Figure 4:** Cell apoptosis in each group in THP-1 cells. Note: ^∗^ indicated that the comparison with NC group showed remarkable difference (*P* < 0.05). # suggested that the comparison with lncRNA GAS5 group demonstrated that the difference showed significant meaning (*P* < 0.05). & revealed that the comparison with Nrf2 group indicated that the difference showed significant meaning (*P* < 0.05).

**Figure 5:** Cell proliferation rate of each group in THP-1 cells. Note: ^∗^ indicated that the comparison with NC group showed remarkable difference (*P* < 0.05). # suggested that the comparison with the lncRNA GAS5 group demonstrated that the difference showed significant meaning (*P* < 0.05). & revealed that the comparison with the Nrf2 group indicated that the difference showed significant meaning (*P* < 0.05).

RETRACTED

**Figure 6:** Results of detection of protein expressions by WB.

**Figure 7:** Comparison of protein contents of IGF1R, STAT3, AKT downstream, and MMP9 in cells of different groups. Note: ^∗^ indicated that the comparison with the NC group showed remarkable difference (*P* < 0.05). # suggested that the comparison with the lncRNA GAS5 group demonstrated that the difference showed significant meaning (*P* < 0.05). & revealed that the comparison with Nrf2 group indicated that the difference showed significant meaning (*P* < 0.05).

**Table 1:** Primers used in this study.

	Primers	Gene sequence
Nrf2	Upstream primer	5′-GGCGTTAGAAAGCAT-CCTTCC-3′
	Downstream primer	5′-GCAGAGGGCACACTCAAAGT-3′

lncRNA CAS5	Upstream primer	5′-TGGATTTCGTGGCCCCAGTGCTA-3′
	Downstream primer	5′-TTCATCCTGTTCTTCCTCGGCG-3′

U6	Upstream primer	5′-GAGAGAAGCCGTCGTGT-3′
	Downstream primer	5′TTGCGAAGTGCTTAAACGCA-3′

## Data Availability

The data is available from the corresponding author upon request.
